# GuanXinNing Tablet Attenuates Alzheimer's Disease via Improving Gut Microbiota, Host Metabolites, and Neuronal Apoptosis in Rabbits

**DOI:** 10.1155/2021/9253281

**Published:** 2021-10-28

**Authors:** Feng Zhang, Yanyun Xu, Liye Shen, Junjie Huang, Songtao Xu, Jiaying Li, Zhichao Sun, Jiangmin He, Minli Chen, Yongming Pan

**Affiliations:** ^1^The Second Clinical Medical College, Zhejiang Chinese Medical University, Hangzhou 310053, China; ^2^Institute of Comparative Medicine, Experimental Animal Research Center, Zhejiang Chinese Medical University, Hangzhou 310053, China; ^3^School of Pharmaceutical Sciences, Zhejiang Chinese Medical University, Hangzhou 310053, China; ^4^The First Clinical Medical College, Zhejiang Chinese Medical University, Hangzhou 310053, China; ^5^The First Affiliated Hospital of Zhejiang Chinese Medical University, Hangzhou 310006, China; ^6^Chiatai Qingchunbao Pharmaceutical Co., Ltd., Hangzhou 310023, China

## Abstract

Based on accumulating evidence, Alzheimer's disease (AD) is related to hypercholesterolemia, gut microbiota, and host metabolites. GuanXinNing Tablet (GXN) is an oral compound preparation composed of two Chinese herbs, *Salvia miltiorrhiza* Bge. and *Ligusticum chuanxiong* Hort., both of which exert neuroprotective effects. Nevertheless, the effect of GXN on AD is unknown. In the present study, we investigated whether GXN alters cholesterol, amyloid-beta (A*β*), gut microbiota, serum metabolites, oxidative stress, neuronal metabolism activities, and apoptosis in an AD model rabbit fed a 2% cholesterol diet. Our results suggested that the GXN treatment significantly reduced cholesterol levels and A*β* deposition and improved memory and behaviors in AD rabbits. The 16S rRNA analysis showed that GXN ameliorated the changes in the gut microbiota, decreased the *Firmicutes/Bacteroidetes* ratio, and improved the abundances of *Akkermansia* and *dgA-11_gut_group*. ^1^H-NMR metabolomics found that GXN regulated 12 different serum metabolites, such as low-density lipoprotein (LDL), trimethylamine N-oxide (TMAO), and glutamate (Glu). In addition, the ^1^H-MRS examination showed that GXN remarkably increased N-acetyl aspartate (NAA) and Glu levels while reducing myo-inositol (mI) and choline (Cho) levels in AD rabbits, consequently enhancing neuronal metabolism activities. Furthermore, GXN significantly inhibited oxidative stress and neuronal apoptosis. Taken together, these results indicate that GXN attenuates AD via improving gut microbiota, host metabolites, and neuronal apoptosis.

## 1. Introduction

Alzheimer's disease (AD), mainly manifested by memory and cognitive deterioration, is the most frequent neurodegenerative disease causing dementia in the elderly [1]. In addition to familial AD, sporadic AD (SAD) accounts for approximately 95% of the incidence of AD and is affected by environmental and genetic factors [2]. Currently, approximately 50 million patients have AD worldwide, and this number is predicted to increase to 131 million by 2050 [3]. Thus, AD has become a growing public health problem [1]. Since the main pathological hallmarks of AD are *β*-amyloid (A*β*) deposition and tau hyperphosphorylation, increasing research and development strategies of anti-AD drugs focus on these two processes [3]. However, most drugs have failed in the clinical research phase [3], indicating that other pathways are involved in AD. Moreover, currently clinically used N-methyl D-aspartic acid receptor antagonists, cholinesterase inhibitors, and other AD drugs have limited efficacy with varying degrees of adverse reactions, usually increasing the difficulties associated with clinical medications for clinicians and patients [4, 5]. Therefore, in-depth studies of the mechanism of AD and its alternative treatment strategies are critical.

In recent years, the gut microbiota has attracted increasing attention due to its critical role in AD. The gut microbiota and its metabolites alter colon permeability and the blood–brain barrier and trigger systemic oxidative stress [6]. Meanwhile, some studies have suggested that gut microbiota disorders affect host nutrition, immunity, and metabolism, and participate in the progression of AD by the gut-brain axis [6, 7]. Moreover, patients with AD exhibit endogenous metabolite disorders and decreased neuronal metabolic activities in the brain [8, 9]. Therefore, gut microbiota and host metabolism may be potential targets for AD treatment. Traditional Chinese medicine (TCM) has the characteristics of multiple ingredients, targets, and pathways [10]. As previously reported, some traditional Chinese herbs ameliorate AD by regulating the gut microbiota and endogenous metabolites, suggesting that TCM may exert a significant effect on modulating gut microbiota and host metabolites [11, 12]. GuanXinNing Tablet (GXN) is an oral compound preparation composed of two Chinese herbs, *Salvia miltiorrhiza* Bge. and *Ligusticum chuanxiong* Hort. [13]. According to our previous liquid chromatography-mass spectrometry (LC–MS) analysis, the main constituents of GXN include salvianolic acid B, ferulic acid, and salvianolic acid A [13].

Although GXN exerts multiple pharmacological effects, such as inhibiting platelet aggregation and antioxidant, anti-inflammatory, and vascular endothelium protection activities [13], the effects of GXN on AD remain unclear. In addition, studies have found that *S. miltiorrhiza* Bge., *L. chuanxiong* Hort., and their active ingredients exert neuroprotective effects [14, 15]. Furthermore, the bioactive components of Danshen, such as salvianolic acid A and salvianolic acid B, and Chuanxiong's bioactive components, such as ferulic acid, exert their effects by regulating gut microbiota and host metabolites [16, 17]. Therefore, we speculate that GXN may regulate the gut microbiota and endogenous metabolites and enhance neuronal metabolic activities via the gut-brain axis, thereby ameliorating AD symptoms.

Diet is considered one of the most critical factors affecting gut microbiota and host metabolites, and high-fat or high-cholesterol diets can cause an imbalance of the gut microbiota and metabolites [18]. In addition, hypercholesterolemia is an important risk factor for AD [19]. Compared with rodent AD models (such as APPswe/PS1dE9 double transgenic mice), rabbits produce A*β* peptide lyase, similar to humans [20, 21]. Moreover, rabbits with AD induced by a 2% high-cholesterol diet developed A*β* deposition in the brain and exhibited more than 10 pathological features similar to those of human patients with AD, such as cognitive decline [19]. Additionally, drug interventions were effective in this rabbit AD model [22], indicating that AD rabbits are suitable for SAD research. In the present study, we investigated the effect of GXN on blood lipid levels, behavior, histopathology, gut microbiota, serum metabolites, oxidative stress, neuronal metabolism activities, and apoptosis in this AD rabbit model to explore its ability to ameliorate AD, reveal the possible mechanism of action, and provide experimental evidence for GXN as a treatment to delay the progression of AD.

## 2. Materials and Methods

### 2.1. Establishment and Intervention of AD Rabbit Model

Eighteen male white hair and black eyes (WHBE) rabbits aged 2 to 3 months (2–2.5 kg) were provided by the Xin Jian Rabbit Field (Zhejiang, China). The certificate number is SCXK, 2015-0004. All rabbits were raised in the Experimental Animal Research Center, Zhejiang Chinese Medical University (Zhejiang, China), with the certificate number SYXK (ZHE) 2018-0012. Rabbits were housed on a 12 h light-dark cycle with free access to food and water. All manipulations complied with the Institutional Animal Care and Use Committee (IACUC) of Zhejiang Chinese Medical University (Approval No. 20190930-06). GXN was obtained from Chiatai Qinchunbao Pharmaceutical Co. Ltd. (Hangzhou, China) and has been approved by the China Food and Drug Administration (No. Z20150028). We identified the main constituents of GXN using LC–MS analysis by referring to previous methods [13]. As shown in Figure 1, the most abundant constituents in GXN are salvianolic acid B (peak 9), rosmarinic acid (peak 7), ferulic acid (peak 5), tanshinol (peak 1), chlorogenic acid (peak 3), caffeic acid (peak 4), and salvianolic acid A (peak 10), which are generally consistent with the results reported by Wang et al. [13].

After two weeks of acclimation, the rabbits were randomized into three groups based on weight and total cholesterol level: the NC group (normal chow, *n* = 6), the AD group (2% cholesterol diet, *n* = 6), and the GXN group (2% cholesterol diet + GXN intervention, *n* = 6). The rabbits in the GXN group were orally administered 250 mg/kg GXN daily for 12 weeks. This dose in the study was determined to be optimal based on our preliminary experiments. The experimental design process is shown in Figure 2. After 12 weeks of treatment, all rabbits were dissected after euthanasia.

### 2.2. Memory Behavior Test

Twelve weeks after administration, the rabbits fasted for 12 hours, and then the memory and behavioral abilities were evaluated using previously reported methods [23]. Drinking water and feed were placed at a fixed site in the 5.4 m^2^ rectangular activity area. Training occurred on the day before the test. During the trial, the feed and drinking water were removed from the fixed point, and SMART video tracking system software (v3.0, Panlab, Spain) was used to record the distances traveled by and times to reach the fixed point within 5 minutes of all rabbits.

### 2.3. Detection of Blood Biochemical Parameters

Each rabbit fasted for 12 hours, and blood biochemical parameters were detected in the 12th week using the corresponding kits (Ningbo Medical System Biotechnology Co. Ltd., China). Blood was obtained via the middle auricular artery. Plasma total cholesterol (TC), triglycerides (TG), high-density lipoprotein cholesterol (HDL-C), and low-density lipoprotein cholesterol (LDL-C) levels were detected using a biochemical analyzer (7020, ITACHI, Japan). In addition, serum levels of oxidative stress markers were measured according to the instructions of the superoxide dismutase (SOD) and malondialdehyde (MDA) kits (Jiancheng Bioengineering Institute, Nanjing, China).

### 2.4. Histopathological Examinations

After an intravenous injection of pentobarbital sodium for anesthesia, the rabbits were perfused transcardially with 300 ml of 4°C PBS. The brain tissues and colon tissues were removed, sliced, and fixed with formalin for 24 h. After fixation, sections were dehydrated with a gradient of ethanol solutions, embedded, and sliced. A Hamamatsu Skeleton Scanner (Nanozoomer S210, Hamamatsu, Japan) was used to scan all sections.

A*β* immunohistochemical staining was performed to examine A*β* deposition. Bax staining and Bcl-2 staining were performed to evaluate apoptosis levels. Briefly, the paraffin sections were dewaxed in water, and peroxidase activity was blocked with 3% H_2_O_2_. Then, the sections were incubated with *β*-amyloid (1:100), Bax (1:200), and Bcl-2 (1:200) antibodies (Santa Cruz Biotechnology, USA) at 4°C overnight. Subsequently, all sections were incubated with the secondary antibody (IgG 1:1000) for 1 hour, stained with DAB, and counterstained with hematoxylin. The positive reaction was specifically stained pale yellow or brownish-yellow.

Thioflavin-T staining was conducted to detect the A*β* content in the brain. Briefly, slides were dewaxed, hydrated in ethanol, and incubated with Mayer's hematoxylin for five minutes. Then, the sections were washed with DW two times and stained with 1% thioflavin-T (Dalian Meilun Biological Technology Co. Ltd., China) for 10 min. After three washes with DW, fluorescence was excited, and the sections were scanned.

IPP 6.0 software was used to analyze the percentages of A*β*-positive and thioflavin-T-positive areas in the entire visual field of the frontal cortex and hippocampus.

Alcian blue and periodic acid-S chiff (AB-PAS) staining were performed to observe colonic epithelial barrier function. The mucus-secreting goblet cells per colonic crypt were stained blue. Briefly, paraffin sections were dewaxed in water, dyed with Alcian blue for 20 min, oxidized in periodic acid for 5 min, and depigmented with Schiff reagent for 20 min. Then, the sections were rinsed, counterstained with hematoxylin, placed in an acidic differentiation solution to induce differentiation, and counterstained blue using Scotts bluing reagent. The AB-PAS positive cells in each crypt from each rabbit in the three groups were counted in five different areas per section. All counts were performed by two independent observers.

### 2.5. 16S rRNA Gene Sequencing and Data Analysis

Twelve weeks after administration, samples of the colon contents were obtained from all rabbits and stored at −80°C, with five samples per group. Total DNA was extracted from the colon contents, and the extraction quality was assessed using agarose gel electrophoresis. Subsequently, the amplicons of the V3–V4 variable region of the 16S rRNA were amplified with specific primers 341F (5′-CCTACGGGNGGCWGCAG-3′) and 805R(5′-GACTACHVGGGTATCTAATCC-3′). 16S rRNA sequencing library was constructed, and 2 × 250 bp paired-end sequencing was performed using a NovaSeq sequencer with the assistance of Hangzhou Lianchuan Biotechnology Co. Ltd. Cutdapt 1.9 software was used to filter low-quality data from the raw sequencing data to ensure the accuracy of the subsequent analysis. FLASH 1.2.8 software was used for double-end splicing, and the double-end data were merged into a long amplicon fragment. Then, the QIIME2 DADA2 plug-in was used for sequence quality control and feature table construction, the QIIME 2 feature-classifier (2019.7) was used for sequence alignment, and the species annotation databases SILVA (release 132) and NT-16S (2019.04.05) were used to perform annotations. Alpha diversity (Chao1 and Shannon) and beta diversity were analyzed. The relative abundances of phyla and genera were compared using Welch's *t*-test in STAMP software. The Kruskal–Wallis test was used to statistically analyze the microbial components, and then the linear discriminant effect size (LEfSe) analysis was performed with the unpaired Wilcoxon test (available from https://huttenhower.sph.harvard.edu/galaxy/).

### 2.6. ^1^H-NMR and Data Analysis

The thawed serum samples (450 *μ*L) and D2O (350 *μ*L) were added to an EP tube. The mixture was vortex mixed thoroughly and centrifuged at 13,000 rpm for 20 min at 4°C. The supernatant (600 *μ*l) was transferred to an NMR tube with a diameter of 5 mm, and NMR spectra were recorded by a Bruker Avance II NMR spectrometer (Bruker BioSpin, Germany). ^1^H-NMR free induction decay (FID) signals were input into Chenomx NMR Suite version 7.7 software (Chenomx, Edmonton, Canada), and automated Fourier transform, phase, and baseline corrections were performed. The ^1^H-NMR map phase and baseline were adjusted using MestReNova 14 (Mestrelab Research, Santiago deCompostella, Spain). The DSS-d6 peak (0.0 ppm) was regarded as the internal standard of all chemical shifts; deconvolution was conducted; and all peak shapes were adjusted. According to the relevant information of the signal in the ^1^H-NMR spectrum, the concentration and peak area of DSS-d6 were used as the standards to normalize the integrated data. Then, we saved the resulting data in an Excel file for further analysis. SIMCA-P14.1 (Umetrics, Umeå, Sweden) was applied to centralize and normalize the integral data. Partial least squares–discriminant analysis (PLS-DA) was performed to observe the dispersion between groups. A permutation test (200 times) was conducted to verify the effectiveness of the PLS-DA model, and orthogonal partial least squares–discriminant analysis (OPLS-DA) was conducted to identify the differentially produced metabolites between samples.

### 2.7. Brain ^1^H-MRS Examination

After 12 weeks of administration, proton magnetic resonance spectroscopy (^1^H-MRS) scanning was performed on a 3.0T MRI scanner. Point resolved spectroscopy (PRESS) was used in ^1^H-MRS scanning. LC Model (Provencher SW, version 6.3) was used to analyze the spectra. The metabolites to be observed in the rabbit brain included the changes in N-acetylaspartic acid (NAA), glutamate complex (Glx), choline (Cho), and myo-inositol (mI) levels, all of which were standardized to creatine (Cr) levels. All operations were performed according to previous research methods [24, 25]. The frontal cortex and hippocampus in the brain were the regions of interest (ROI; Figure 3(a)).

### 2.8. TUNEL Staining of Brain Tissues

We determined neuronal apoptosis by conducting a TUNEL assay according to the instructions provided with the corresponding kits (Baori Medical Biotechnology Co. Ltd., China). Images of six randomly selected visual fields of the cortex and the hippocampus (three fields for each region) were captured. TUNEL-positive cells were stained green, and nuclei were stained blue. The number of positive cells and the total number of neurons per field were counted, and the apoptosis index (AI; AI = number of positive cells/total number of neurons) was calculated.

### 2.9. Statistical Analysis

Data are presented as means ± SEM. GraphPad Prism 8.0 software (GraphPad Software, Inc., La Jolla, CA, USA) was applied for statistical analyses using one-way ANOVA with Tukey's post hoc test (^*∗*^*P* < 0.05 and ^*∗∗*^*P* < 0.01 versus the AD model group). Pearson's correlation coefficient (*R*) was calculated to analyze correlations. *P* < 0.05 was considered statistically significant.

## 3. Results

### 3.1. GXN Reduced Blood Lipid Levels, Improved Memory and Behaviors, and Alleviated A*β* Pathology in the Brains of AD Rabbits

As shown in Figure 4(a), the GXN group showed 31.6% and 37.8% reductions in plasma levels of TC and LDL-C compared to the AD group, respectively (*P* < 0.01). In addition, the body weight of the three groups did not change significantly (*P* > 0.05). Furthermore, the memory and behavioral tests suggested that the distance traveled and time to reach a fixed point in the AD group were significantly prolonged compared with those in the NC group (*P* < 0.01). In contrast, GXN treatment significantly reduced the distance traveled and time by 69.6% and 57.4%, respectively (*P* < 0.01; Figures 4(b) and 4(c)). In addition, A*β*-staining showed significantly decreased A*β* expression in both the cortex and hippocampus of the GXN group relative to the AD group (*P* < 0.01; Figures 4(d) and 4(e)). Moreover, thioflavin-T staining showed that the GXN intervention significantly reduced the plaque-covered areas in both the cortex and hippocampus compared to the AD group (*P* < 0.01; Figures 4(f) and 4(g)).

### 3.2. GXN Improved Colon Barrier Permeability and the Diversity of Gut Microbiota in AD Rabbits

As a dynamic semipermeable barrier, the gut mucus layer is a vital component of the colon barrier. In the NC group, the epithelial cells and goblet cells in the colonic mucosal layer exhibited a normal morphology, and abundant mucus secretion on the mucosal surface was observed, whereas in the AD group these cells showed variable degrees of atrophy and mucus secretion decreased (Figure 5(a)). Compared with the AD group, the epithelial cells and goblet cells at various levels of recovery were observed in the GXN group, and mucus secretion also increased. Quantitatively, the GXN intervention significantly increased the number of AB-PAS-positive cells per crypt (*P* < 0.05; Figure 5(b)). In addition, *α*-diversity is a composite indicator used to assess species evenness and richness in a single community sample. The Chao1 index mainly reflects the abundance of species in the sample, and the Shannon index mainly reflects the diversity of species in the community. Compared with the NC group, the Chao1 index in the AD group was slightly increased (Figure 5(c); *P* > 0.05), while the Shannon index was significantly increased (Figure 5(d); *P* < 0.05). Nevertheless, in the GXN group, the Chao1 index was slightly decreased compared to that in the AD group (*P* > 0.05), while the Shannon index was significantly decreased (*P* < 0.05). *β*-Diversity reflects changes in the gut microbiota structure among different samples. As shown in Figure 5(e), principal coordinate analysis (PCoA; *P*=0.004) suggested that the AD group significantly deviated from the NC group, and the GXN group was nearer to the NC group than the AD group.

### 3.3. GXN Improved the Structure of the Gut Microbiota in AD Rabbits

Eleven major phyla were identified in the gut microbiota of WHBE rabbit colon contents, including *Firmicutes*, *Bacteroidetes*, and *Verrucomicrobia* (Figure 6(a)). Compared with the AD group, the GXN intervention significantly decreased the *Firmicutes*/*Bacteroidetes* ratio and the abundance of *Firmicutes* (*P* < 0.05 and *P* < 0.01; Figures 6(b) and 6(c)) and significantly increased the abundance of *Verrucomicrobia* (*P* < 0.05; Figure 6(c)), indicating that GXN ameliorated gut microbiota disorders.

The classification level was further refined to the genus level, and the top 20 genera are listed in Figure 6(d). In the comparison of the AD and NC groups, 10 bacterial genera were significantly changed (*P* < 0.05 and *P* < 0.01; Figure 6(e)), including *Akkermansia*, *Firmicutes_unclassified*, and *dgA-11_gut_group*. Meanwhile, in the comparison of the GXN and AD groups, the abundance of five bacterial genera (*Akkermansia*, *dgA-11_gut_group*, *Ruminiclostridium_5*, *Intestinimonas*, and *Moryella*) was significantly altered (*P* < 0.05). Furthermore, an LEfSe analysis was conducted using the Galaxy version 1.0.0 online analysis tool to further determine the bacteria targeted by GXN. The biomarkers of the gut microbiota on the evolutionary branch at each level of classification were detected. The results further confirmed that *Akkermansia* and *dgA-11_gut_group* were significantly affected in the AD rabbit, and the GXN intervention significantly regulated the abundance of these bacteria (Figure 6(f)), suggesting that *Akkermansia* and *dgA-11_gut_group* may be the target bacterial genera of the anti-AD effects of GXN.

Pearson's correlation analysis was conducted to assess the correlations between representative gut microbiota, blood lipid levels, A*β*, and neuronal metabolism activities in AD rabbits. As shown in Figure 6(g), TC, LDL-C, and A*β* levels in the hippocampus and cortex, and mI and Cho levels were positively associated with the *dgA-11_gut_group* (*P* < 0.05 and *P* < 0.01), while Glx and NAA levels showed a negative correlation (*P* < 0.01). In addition, *Akkermansia* was negatively correlated with TC, LDL-C, A*β*, and mI levels (*P* < 0.05).

### 3.4. GXN Altered Serum Metabolite Levels in AD Rabbits

Twenty-four endogenous metabolites were identified by analyzing the characteristics of the spectra and combining them with the NMR data available in the literature and the Human Metabolome Database (HMDB, http://www.hmdb.ca/) [10]. The typical ^1^H-NMR spectrum of each group and metabolites identified are shown in Figure 7.

Multivariate statistical analysis and visualization were performed to more visually observe the changes in metabolites in AD rabbits and the improvement effect of administration of GXN. The PLS-DA score plot (Figure 8(a); *R*^2^*X* = 0.915, *R*^2^*Y* = 0.832, and *Q*^2^ = 0.619) showed that the three groups were separated, indicating that the metabolites in the AD rabbits were disordered after modeling and that the GXN intervention regulated the metabolites in AD rabbits. Then, a permutation test (*n* = 200) was subsequently conducted to validate the PLS-DA and avoid overfitting. As shown in Figure 8(b), the permutation test suggested that the PLS-DA model had appropriate *R*^2^*Y* (0, 0.44) and Q^2^ (0, −0.249) values, suggesting that the PLS-DA model was not overfitted and had good prediction ability.

Furthermore, OPLS-DA was conducted between the AD and GXN groups to determine the differentially altered metabolites. Consistent with the results of the PLS-DA score plot, the OPLS-DA model (Figure 8(c); *R*^2^*X* = 0.787, *R*^2^*Y* = 0.994, and *Q*^2^ = 0.953) also suggested a separation between the AD and GXN groups. Furthermore, based on the *P* values (*P* < 0.05; ANOVA) and VIP values (VIP  > 1), 12 differentially altered metabolites were screened (Figure 8(d)). Compared with the AD group, the serum LDL, glycerol, glycine, TMAO, and creatine levels in the GXN group were significantly decreased (*P* < 0.05 and *P* < 0.01), while leucine, isobutyric acid, valine, glutamate, 3-hydroxybutyrate, acetic acid, and citric acid levels were significantly increased (*P* < 0.05 and *P* < 0.01), suggesting that GXN may ameliorate AD by regulating the levels of these metabolites. Finally, the 12 differentially altered metabolites mentioned above were imported into MetaboAnalyst 5.0 software (https://www.metaboanalyst.ca/) for a pathway enrichment analysis to identify the key metabolic pathways related to the effect of GXN on ameliorating AD. Seven metabolic pathways (whose *P* < 0.05 or Impact >0.1) related to the effect of GXN on ameliorating AD were obtained (Figure 8(e)).

### 3.5. GXN Improved Neuronal Metabolism Activities in AD Rabbits

^1^H-MRS was performed to evaluate the alterations of neuronal metabolism activity in the rabbit brain, and the metabolites from ^1^H-MRS spectra were identified in Figure 3(b). Quantitatively, in the AD group, the NAA/Cr and Glx/Cr levels in the brain were significantly reduced compared to those in the NC group (*P* < 0.01; Figure 3(c)), whereas the Cho/Cr and mI/Cr levels were significantly increased (*P* < 0.01). In contrast, GXN treatment produced 19.1% and 31.0% increases in the NAA/Cr and Glx/Cr levels, respectively (*P* < 0.05), and 31.3% and 18.3% reductions in the Cho/Cr and mI/Cr levels, respectively (*P* < 0.05 and *P* < 0.01).

### 3.6. GXN Inhibited Apoptosis-Related Protein Expression and Enhanced Antioxidant Capacities in AD Rabbits

The expression of the Bax and Bcl-2 proteins was observed in the immunohistochemistry images. The nucleus was stained blue, and the positive staining was brown (Figures 9(a) and 9(c)). In the GXN group, Bcl-2 expression in the cortex and hippocampus was remarkably increased (*P* < 0.05), while Bax expression was remarkably decreased relative to that in the AD group (*P* < 0.05 and *P* < 0.01; Figures 9(b) and 9(d)). Furthermore, in the GXN group, the Bax to Bcl-2 ratio in the brain was significantly decreased compared to that in the AD group (*P* < 0.01; Figure 9(e)). In addition, the GXN intervention remarkably increased SOD levels (*P* < 0.01) and significantly reduced MDA levels (*P* < 0.05; Figure 9(f)).

### 3.7. GXN Attenuated Neuronal Apoptosis in AD Rabbits

A TUNEL assay was conducted to observe neuronal apoptosis in rabbits. As shown in Figure 10, the AI of the cortex and hippocampus was significantly increased in the AD group compared to the NC group (*P* < 0.05), whereas the GXN intervention significantly decreased the AI of the cortex and hippocampus (*P* < 0.01).

## 4. Discussion

Our study confirmed that a high-cholesterol diet induced some typical AD symptoms and AD pathological manifestations in a rabbit model. In contrast, GXN treatment decreased the TC and LDL levels, the *Firmicutes*/*Bacteroidetes* ratio, and the abundance of *dgA-11_gut_group*; increased the abundance of *Akkermansia*; and improved serum and brain metabolite disorders. Meanwhile, GXN also increased SOD and Bcl-2 levels, decreased MDA and Bax levels, and ameliorated A*β* deposition, neuronal apoptosis, and memory deficits in AD rabbits induced by a high-cholesterol diet. Based on our results, GXN attenuated AD.

Hypercholesterolemia is a significant risk factor for AD and was proven to enhance the activity of the *β*-secretase pathway that processes amyloid precursor protein through the formation of lipid rafts, thereby promoting A*β* deposition, aggravating A*β* neurotoxicity, and subsequently leading to the occurrence of AD [26]. In addition, previous studies have suggested that hypercholesterolemia is closely related to cognitive decline [27]. Clinically, patients with AD are characterized by progressive memory and cognitive decline [28]. These characteristics are consistent with the changes in the AD model rabbits fed a 2% cholesterol diet. In contrast, the GXN intervention significantly reduced TC and LDL-C levels, inhibited brain A*β* deposition, and improved memory and behaviors in AD rabbits. Thus, GXN may inhibit A*β* deposition and memory and behavioral deficits by reducing cholesterol levels in AD rabbits.

Based on accumulating evidence, the gut microbiota and its metabolites affect AD; consequently, the gut microbiota is also considered a potential therapeutic target for AD [29, 30]. AB-PAS staining evaluates the integrity of colonic epithelial barrier function [31]. Goblet cells secrete mucin, which covers the surface of the colonic mucosa to form a mucus barrier and maintain the integrity of the colonic barrier [32]. In addition, 16S rRNA sequencing evaluates the changes in the gut microbiota structure to further reveal other potential mechanisms by which GXN ameliorates AD. Previous studies have found that a high-cholesterol diet causes gut microbiota dysbiosis, damage to colonic barrier integrity, and host metabolic disorders [18, 33]. Similarly, changes in gut microbiota diversity and a decreased number of mucus-secreting goblet cells per colonic crypt were observed in our study. In contrast, GXN significantly ameliorated gut microbiota diversity and increased the number of goblet cells, suggesting that GXN may exert its effect by improving the gut microbiota and colon barrier permeability. In addition, GXN remarkably increased the abundance of *Akkermansia* and decreased the abundance of the *dgA-11_gut_group* in AD rabbits. *Akkermansia* is a representative genus in the human gut microbiota in the *Verrucomicrobia* phylum, and a high-fat diet can reduce its abundance [34]. As previously reported, *Akkermansia* preserves colonic barrier permeability, reduces blood endotoxin levels, improves insulin resistance, and protects AD model mice from cognitive deficits and amyloid pathology, indicating that it may slow the progression of AD [35]. In addition, as a bacterium that produces short-chain fatty acids (SCFAs) [36], a decrease in the level of *Akkermansia* was also considered to cause inflammation, impaired glucose tolerance, and diet-induced obesity [37], thereby participating in the development of AD. In addition, the *dgA-11_gut_group* was proposed to be related to lipid metabolism disorders, which are vital factors contributing to AD [38]. Furthermore, the LEfSe analysis confirmed that *Akkermansia* and the *dgA-11_gut_group* might be the target bacteria of the anti-AD effects of GXN, and a subsequent correlation analysis showed that *Akkermansia* and the *dgA-11_ gut_ group* were significantly correlated with AD-related clinical indices. Therefore, these results indicated that GXN may exert an anti-AD effect by regulating *Akkermansia* and the *dgA-11_gut_group* and ameliorating gut microbiota dysbiosis.

^1^H-NMR metabolomics and pathway enrichment analyses showed that the GXN intervention significantly reduced LDL and TMAO levels in AD rabbits, increased glutamate, citric acid, 3-hydroxybutyric, and leucine levels and was involved in D-glutamine and D-glutamate metabolism and glutathione metabolism. Glutamate, a precursor for the synthesis of the natural antioxidant glutathione (GSH), is presumed to play a vital role in cellular antioxidant defenses [39]. GSH prevents oxidative damage and neuronal apoptosis by reducing H_2_O_2_ levels, thereby delaying the progression of AD [39]. In addition, TMAO (a gut microbiota-related metabolite) levels are significantly increased in patients with AD and positively correlate with AD markers (A*β* and p-tau) [40]. Citric acid is a significant intermediate product of the tricarboxylic acid cycle and the hub of the metabolic connection of lipids [41]. Leucine and 3-hydroxybutyric acid affect lipid metabolism and synthesis and intrahepatic mitochondrial lipid metabolism [42, 43]. Thus, GXN may ameliorate AD by inhibiting lipid synthesis and reducing lipid peroxidation and neuronal apoptosis.

Furthermore, ^1^H-MRS indicated that GXN significantly enhanced neuronal metabolism activities, such as increasing Glx/Cr and NAA/Cr levels and decreasing Cho/Cr and mI/Cr levels. Studies have shown that metabolic changes in the brain are significantly related to cognitive decline, and the symptoms of dementia in patients with AD are postulated to be associated with a decline in neuronal metabolic activities [8, 9]. Therefore, an abnormal metabolic function in the brain is considered a critical pathological factor that causes AD [44]. NAA is a specific biomarker of the severity of the neuronal injury, and its level is significantly decreased in patients with AD [45]. Glx is the most abundant excitatory neurotransmitter in the brain and has multiple functions in the nervous system [46]. Decreased levels of Glx reflect the loss or decreased activity of glutamatergic neurons, which is a significant pathological feature in the brains of patients with AD. In addition, Cho is one of the components of cell membrane phospholipid metabolism and is involved in the synthesis and metabolism of cell membranes [47]. mI participates in astrocyte activation and proliferation and is a significant marker indicating the severity of inflammation in the brain [48]. Thus, GXN may stabilize nerve cell membranes, inhibit the activation of glial cells, and improve neuronal metabolism in AD rabbits, thereby ameliorating AD.

In addition, under normal physiological conditions, reactive oxygen species (ROS) are eliminated by the antioxidant substances in the body [49]. Hypercholesterolemia, gut microbiota dysbiosis, and destruction of the colon barrier are related to oxidative stress [50, 51]. In individuals with AD, A*β* neurotoxicity and oxidative stress damage neurons by inducing apoptosis [26, 52], thereby leading to cognitive decline [53]. In our study, the GXN intervention significantly reduced the A*β* load in AD rabbits. Furthermore, four markers were examined to evaluate oxidative stress and the changes in apoptotic activities: SOD (a free radical scavenger used to evaluate the generation of free radicals), MDA (a sensitive indicator of the strength of oxidative stress), and Bax and Bcl-2 (vital regulatory genes involved in cell apoptosis). Bax promotes apoptosis, while Bcl-2 inhibits apoptosis. The Bax to Bcl-2 ratio determines the degree of apoptosis: the higher the ratio, the greater the apoptosis. Our study suggested that GXN remarkably suppressed oxidative stress and apoptosis-related protein expression. Moreover, the TUNEL assay also indicated that the GXN intervention significantly ameliorated apoptosis in the cortex and hippocampus. Based on these results, GXN may have the potential to prevent neuronal apoptosis by suppressing A*β* neurotoxicity, oxidative stress, and Bax expression and promoting Bcl-2 expression.

However, our study had some limitations. First, although the reliability of the rabbit AD model and the effectiveness of drug interventions have been reported, the present study did not include a positive reference drug group, which may not fully reflect the advantages of GXN. Second, although the characteristic metabolite changes induced by GXN to ameliorate AD were obtained using ^1^H-NMR, some other potential metabolites may be omitted due to the limited number of metabolites detected using this method. Therefore, the design of positive reference drugs and detection of metabolites using q-TOF/MS or Orbitrap-based methods are necessary to further evaluate the efficacy and mechanism of action of GXN in AD.

## 5. Conclusion

In conclusion, our current study suggested that GXN ameliorated AD symptoms by reducing cholesterol levels and A*β* deposition, regulating disorders of gut microbiota and serum metabolites, enhancing neuronal metabolic activities, and inhibiting oxidative stress and neuronal apoptosis (Figure 11). Together, these results reveal the possible mechanisms by which GXN ameliorates AD, providing experimental evidence that GXN delays AD progression.

## Figures and Tables

**Figure 1:** LC–MS chromatogram of GXN: (1) tanshinol, (2) protocatechualdehyde, (3) chlorogenic acid, (4) caffeic acid, (5) ferulic acid, (6) senkyunolide I, (7) rosmarinic acid, (8) isosalvianolic acid A, (9) salvianolic acid B, and (10) salvianolic acid A.

**Figure 2:** Flow chart of the study.

**Figure 3:** GXN improved rabbit neuronal metabolism activities: (a) the white box indicates the ROI in the brain, (b) the metabolites in ^1^H-MRS spectra were identified, and (c) changes in metabolites in each group (*n* = 6).

**Figure 4:** GXN reduced blood lipid levels, improved memory and behaviors, and alleviated A*β* deposition in the brains of AD rabbits. (a) The effects of GXN on body weight and TC, TG, HDL-C, and LDL-C levels in AD rabbits. (b) Representative traces of the path traveled by each group in the memory and behavior test. (c) Quantitative analysis of the distance traveled and time to reach a fixed point of each group. (d, f) Representative images of A*β* and thioflavin-T staining in each group. Scale bar = 50 mm. White or black boxes indicate the region shown at higher magnification below each panel. (e, g) Quantitative analysis of A*β* levels and plaque-covered area in each group. *n* = 6.

**Figure 5:** GXN improved colon barrier permeability and the diversity of gut microbiota in AD rabbits. (a) Typical images of AB-PAS staining in the colon tissue. Scale bar = 500 mm. Black boxes indicate the areas shown at higher magnification. (b) Quantitative analysis of the number of AB-PAS-positive cells per crypt in each group. Chao1 (c) and Shannon (d) indices of *α*-diversity were assessed. (e) Principal coordinate analysis (PCoA) of the *β*-diversity index. *n* = 5.

**Figure 6:** GXN improved the structure of the gut microbiota in AD rabbits: (a) and (d) relative abundance at the phylum and genus levels; (b) the *Firmicutes/Bacteroidetes* ratio; (c) and (e) changes in specific phyla and genera; (f) evolutionary branch diagrams comparing the gut microbiota in the AD and GXN groups; and (g) heatmap of Pearson's correlation coefficients between representative components of the gut microbiota, blood lipids, A*β*, and neuronal metabolism activities. *n* = 5. Red and blue indicate positive correlations and negative correlations, respectively.

**Figure 7:** Representative ^1^H-NMR spectra from rabbits: (a) the NC group, (b) the AD group, and (c) the GXN group. (1) LDL, (2) leucine, (3) isoleucine, (4) valine, (5) isobutyric acid, (6) 3-hydroxybutyrate, (7) lactate, (8) alanine, (9) lysine, (10) Acetic acid, (11) glutamate, (12) pyruvate, (13) glutamine, (14) citric acid, (15) TMA, (16) creatine, (17) creatinine, (18) TMAO, (19) betaine, (20) proline, (21) glycerol, (22) L-carnitine, (23) glycine, and (24) glucose.

**Figure 8:** GXN altered serum metabolite levels in AD rabbits: (a) PLS-DA score plot for each group, (b) permutation test of the PLS-DA model, (c) OPLS-DA score plot of the AD group versus the GXN group, (d) relative serum contents of different metabolites in rabbits from each group, and (e) schematic representation of pathways identified by MetaboAnalyst 5.0. The ordinate indicates the significance level of the metabolic pathway, and the abscissa indicates the importance of the metabolic pathway. (1) D-glutamine and D-glutamate metabolism; 2. glycine, serine, and threonine metabolism; 3. glycerolipid metabolism; 4. alanine, aspartate, and glutamate metabolism; 5. glyoxylate and dicarboxylate metabolism; 6. arginine biosynthesis; and 7. glutathione metabolism. *n* = 6. Red and blue indicate positive correlations and negative correlations, respectively.

**Figure 9:** GXN inhibited apoptosis-related protein expression and enhanced serum antioxidant capacities. Representative images of Bax (a) and Bcl-2 staining (c) in three groups of rabbits. Scale bar = 50 mm. Black boxes indicate the areas shown at higher magnification. Quantitative analysis of percentages of Bax-positive staining (b) and Bcl-2-positive staining (d) in each group. (e) Bax/Bcl-2 ratio in each group. (f) Changes in serum SOD and MDA levels in each group. *n* = 6.

**Figure 10:** GXN attenuated neuronal apoptosis in AD rabbits. (a) Representative images of TUNEL staining in the three groups of rabbits. Scale bar = 50 mm. (b) Quantitative analysis of the percentage of TUNEL-positive cells in each group. *n* = 6.

**Figure 11:** Schematic diagram of possible mechanisms by which GXN ameliorates AD in high-cholesterol diet-induced rabbits. GXN reduces cholesterol levels, the *Firmicutes/Bacteroidetes* ratio, and the abundance of *dgA-11_gut_group*; increases the abundance of *Akkermansia*; and attenuates serum and brain metabolite disorders. Meanwhile, GXN also increases SOD levels, decreases MDA levels, and attenuates A*β* deposition and neuronal apoptosis, thereby ameliorating AD symptoms in rabbits fed a high-cholesterol diet. Arrows indicate statistically significant increases and decreases (*P* < 0.05). The red and green arrows suggest the changes in AD model rabbits and the therapeutic effects of GXN, respectively.

## Data Availability

The data are available from the corresponding author on reasonable request.
